This article has been retracted.

# Three-Dimensional Mapping of Medial Wall in Unstable Pertrochanteric Fractures

**DOI:** 10.1155/2020/8428407

**Published:** 2020-05-31

**Authors:** Yingqi Zhang, Yeqing Sun, Shenghui Liao, Shimin Chang

**Affiliations:** ^1^Department of Orthopedic Surgery, Tongji Hospital, Tongji University School of Medicine, Shanghai, China; ^2^School of Information Science and Engineering, Central South University, Changsha, China; ^3^Department of Orthopedic Surgery, Yangpu Hospital, Tongji University School of Medicine, Shanghai, China

## Abstract

**Objective:**

Unstable pertrochanteric fractures are usually treated with internal fixation, and the integrity of the anteromedial cortex is an important factor for stability and healing. In this study, we described and analyzed the three-dimensional mapping technology and morphological characteristics of pertrochanteric fractures.

**Methods:**

Fifty-nine pertrochanteric fractures (OTA/AO 2007 types 31A2) were retrospectively reviewed. Computed tomographic (CT) images for all fractures were superimposed on a standard template. Medial wall integrity was analyzed, and three-dimensional fracture maps were created.

**Results:**

Pertrochanteric fractures always have a posterior defect in the medial cortex. The mean width of the defect, in our study, was 21.5 mm (SD: 6.1 mm, range: 10–40 mm), 56.3% (SD: 13.7%, range: 27.5-100%). Bone segments that contact by the anteromedial cortex were 16.5 mm (SD: 5.3 mm, range: 0-29 mm).

**Conclusion:**

The integrity of the anteromedial cortex should be considered during internal fixation of femoral trochanteric fractures. These morphological characteristics could be used to form postoperative cortical contact and improve stability of the fixation. Three-dimensional mapping technology can help establish a typical fracture model, thereby improving doctors' understanding of fracture characteristics.

## 1. Introduction

Pertrochanteric femoral fractures constitute a significant proportion of hip injuries, which continues to be a challenge for orthopedic trauma surgeons in daily practice. The integrity of the medial cortex has gained increasing focus to address issues concerning the stability of reconstructions after fracture fixation [1, 2]. It affects internal fixation stability and fracture prognosis [3].

Fracture mapping is a method for describing the morphology of bone fractures proposed by Armitage et al. [4] in 2009. This technique can reveal the frequency of fracture lines, the type of bone fracture, and the degree of comminution and articular surface defects. The 2-dimensional fracture mapping technique was first described by Cole et al. [5]. This technique has been applied to characterize pilon and scapular fractures. Molenaars et al. combined mapping with 3D bone reconstruction and reduction for characterizing the tibial plateau and articular surface of the radial head fracture [6]. However, a previous study was based on the two-dimensional (2D) fracture lines and separate fracture fragments that were mapped. In this study, 3D mapping of the fracture lines and bone defects was established. While more studies are devoted to the use of fracture mapping in fractures of the articular surface, few reports have been published on its application in fractures of the nonarticular surfaces.

However, the three-dimensional morphological characteristics of pertrochanteric fractures are not clear. In this study, we summarized fracture information by utilizing a new three-dimensional (3D) mapping technology. This study describes an improved 3D fracture mapping technique with morphological characterization of pertrochanteric fractures. We hope to enhance the understanding of pertrochanteric fractures by establishing a standard model to aid the biomechanical modeling and clinical process.

## 2. Patients and Methods

### 2.1. Patient Cohort and Fracture Classification

The retrospective design was approved by the ethics committee. One hundred and thirty patients with pertrochanteric fractures were diagnosed by radiography in two centers, from January 2017 to October 2018. In total, 101 cases that had CT scan data were selected. All CT assessments were performed using a 64-slice spiral computed graphic scanner (General Electric Company, American). Scanning parameters were set as follows: 120 kV, 350 mA, 0.625 mm thickness, and 1 s rotation time. Scanning was performed from the anterior superior iliac spine to the femoral lesser trochanter. Based on CT reconstruction, the fracture was subjected to OTA classification. Only those fractures confirmed by CT as OTA type A2 were included for the analysis of medial wall integrity and 3D mapping. Data from A2 cases underwent processing as described below.

### 2.2. Distribution of the Separate Fracture Fragments

The entire femur trochanter area was divided into six parts: anteromedial region, posteromedial region, pertrochanteric crest, greater trochanter, lateral wall, and pertrochanteric line. The number of separate fracture fragments in each position was counted.

### 2.3. Three-Dimensional Fracture Mapping

The procedures of 3D mapping are presented in Figures 1 and 2.

#### 2.3.1. 3D Reconstruction and Reduction

All CT data were fed into the Boholo medical imaging software (E-3D, Changsha, China) to reconstruct the 3D proximal femur osseous structure. All separate fracture fragments were created as a 3D polygon mesh model, and a virtual reduction was performed for the separate fracture fragments (Figures 1(a)–1(c)).

#### 2.3.2. Tracing the Fracture Lines on the 3D Model Surface

The model of a normal proximal femur was taken as the standard. Using the software, the fracture lines were mapped to the standard model for each case, and the separate fracture fragments were defined (Figures 1(e)–1(g)).

#### 2.3.3. Fracture Line Superposition

The fracture lines of all cases were represented in the standard model to obtain the distribution map of the fracture lines (Figures 2(a)–2(e)).

#### 2.3.4. Frequency Heat Mapping of Fracture Lines

The fracture line area was defined as the area within 2 mm from the fracture line. The closer the distance to the fracture line, the higher the weight assigned to the fracture line. Thus, the fracture lines of all cases were superimposed to calculate the frequency of fracture lines in the 3D model. In heat maps, the relative fracture line distribution (e.g., fracture line intensity) was represented as color following arbitrary units of measurement (Figures 3(a)–3(e)).

#### 2.3.5. Fracture Location Mapping

The head-neck and shaft fragments were the major fragments after reduction. Other fracture fragments such as the lesser trochanter, greater trochanter, and pertrochanteric crest were considered as bone defects. The defect fragment locations in all cases were superimposed to calculate the frequency distribution of fracture locations (Figures 4(a)–4(e)).

#### 2.3.6. Support Line Mapping

For patients with OTA type A2 fractures, stability was mainly offered by the contact between the fracture fragments in the femoral head-neck and shaft. In this study, the support lines were analyzed separately to observe the support features (Figures 5(a)–5(e)).

### 2.4. Integrity of Medial Wall

After simulating reduction, in the medial view (perpendicular to neck axis), five parameters were recorded (Figure 1(d)): (a) medial wall width (Mww), (b) defect width (Dw), (c) connected medial wall width (Cmww), (d) distance between defect and neck axis (Dd), and (e) ratio between Cmww and Mww.

## 3. Results

A total of 101 cases with a greater trochanter fracture were collected, of which four cases showed a simple greater trochanteric fracture and 97 showed intertrochanteric and pertrochanteric fractures. These 97 cases were further classified.

### 3.1. OTA/AO Classification

There were 21 cases of proximal femoral pertrochanteric simple (only two fragments) fractures (31-A1): nine cases with type A1.1 fracture, six cases with type A1.2 fracture, and six cases with type A1.3 fracture.

There were fifty-nine cases of proximal femoral pertrochanteric multifragmentary (always having posteromedial fragment with lesser trochanter and adjacent medial cortex) fractures (31-A2): 15 cases with type A2.1 fracture, 28 cases with type A2.2 fracture, and 16 cases with type A2.3 fracture.

There were seventeen cases of proximal femoral fracture, trochanteric fracture, or pertrochanteric fracture (31-A3): two cases with type A3.1 fracture, five cases with type A3.2 fracture, and 10 cases with type A3.3 fracture.

The locations of the fracture surface were analyzed and mapped for 59 OTA/AO type A2 fractures. Of these patients, the mean age was 64 (range, 42–79) years. There were 38 (64%) men and 21 (36%) women.

### 3.2. Distribution of Separate Fracture Fragments

There are six kinds of separate fracture fragments in our study:

1. Posteromedial region: 59 cases (100.00%), 2.03 ± 0.98 fracture fragments on average
2. Pertrochanteric crest: 40 cases (67.80%), 0.83 ± 0.70 fracture fragments on average
3. Greater trochanter: 56 cases (67.80%), 1.61 ± 0.87 fracture fragments on average
4. Lateral wall: 12 cases (20.34%), one fracture fragment in each case
5. Pertrochanteric line: eight cases (13.65%), one fracture fragment in each case
6. Anteromedial region: two cases (3.96%), one fracture fragment in each case

### 3.3. Integrity of Medial Wall

The Mww is 38.0 mm (SD: 4.2 mm, range:28-46 mm), Cmww is 16.5 mm (SD: 5.3 mm, range: 0-29 mm), Dw is 21.5 mm (SD: 6.0 mm, range: 10-40 mm), Cmww/Mww is 43.7% (SD: 13.6%, range: 0.0%-72.5%), and Dd is -3.6 mm (SD: 5.7 mm, range: from -17.0 mm to 15.0 mm). In 16 cases, defect fragments involved the anteromedial area.

## 4. Discussion

An unstable pertrochanteric fracture remains a major challenge for orthopedists owing to its high nonunion rate, high incidence of postoperative complications, low patient satisfaction, and high cost. The morphology of a pertrochanteric fracture is closely related to the clinical efficacy. While CT has facilitated the description of some new imaging characteristics of unstable pertrochanteric fractures, there is still a lack of comprehensive and intuitive summary of the imaging characteristics of this type of bone fracture. In this study, we presented a description of the CT characteristics of an unstable pertrochanteric fracture and its mapping pattern.

### 4.1. 3D Mapping

In 2009, Armitage et al. applied fracture mapping to describe the characteristics of a scapular fracture [4]. Nowadays, this technique has been used in studies regarding morphology of various bone fractures, including pilon, tibial plateau, and radial head fractures [7]. Over the course of time, the focus of attention has shifted from displaying the fracture line distribution [4] to heat mapping of the bone-fracture frequency [7]. The technique used has evolved from CT-based bone reposition [6] to 3D reconstruction [7]. Given the limitations of graphic technologies, 2D mapping of the articular surface or flat bone once dominated. In this study, we used 3D mapping of the unstable pertrochanteric fracture. As 3D heat mapping is impossible for the stereo structure using conventional 2D pixels, we calculated the weight of the distance of fracture lines on the 3D surface and presented a novel 3D heat mapping method to analyze the 3D characteristics of the bone fracture.

### 4.2. Fracture Line Distribution

The fracture line distribution was analyzed statistically and subjected to graphic processing. In the front, the fracture lines mainly extended along the pertrochanteric line; in the rear, the fracture lines were primarily located at the junction between the femoral base and the pertrochanteric crest. The fracture lines in the two parts converged in the anterior region of the lesser trochanter, encircling the lesser trochanter and extending inferiorly.

Among previous efforts in biomechanical modeling, no standard models of trochanteric fracture have yet been established. Some researchers completely removed the medial region of the femur to form a wedge-shaped defect [8–11], while others removed the lesser trochanter fragment that was narrow in the front and wide in the back [10, 12]. Moreover, the medial region has always been completely damaged. We found that the defects were mainly distributed in the posterior half of the medial wall, while the anterior half remained intact. The head-neck segment was still in effective contact with the femoral shaft. This mechanical feature was very important to understand the unstable pertrochanteric fracture, which can be used as the modeling criteria in biomechanical modeling and finite element analysis. During surgery, this contact area could be used to achieve maximum internal fixation stability, as has been verified by a prior study [13].

### 4.3. Support Lines and the Anteromedial Region

Pertrochanteric fractures are mainly treated by extramedullary fixation such as a dynamic hip screw (DHS) or intramedullary fixation such as proximal femoral nail antirotation (PFNA). After fracture reduction and fixation, the movement of the head-neck fragment is mostly guided to slide in an axial direction along the implant (helical blade or lag screw) to the lateral side (telescoping). Limited telescoping provides controlled fracture impaction to achieve secondary axial and torsional stability between the head-neck fragment and femur shaft [13].

The forces caused by weight bearing on the femoral head are transmitted to the femoral shaft by three points through direct bone contact and the bone-implant construct: (1) the implant in the femoral head, (2) the superolateral corner between the neck and later trochanteric wall, and (3) the anteromedial corner between the neck and shaft cortices. As the anteromedial cortex is the only remnant containment that could be used to share the load with the implant, obtaining anteromedial cortex support through the fracture reduction technique is of paramount importance and an effective biological approach to prevent oversliding. The anteromedial cortex of the head-neck fragment should be displaced and located a bit more superomedially (for the medial cortex) and anteriorly (for the anterior cortex) to the cortex of the femur shaft in the anteroposterior and lateral views, as this will allow limited telescoping of the head-neck fragment postsurgery to contact with the femur shaft and achieve secondary stability. Meanwhile, cortical contact between the two main fragments is achieved, and the anteromedial cortex of the femoral shaft can resist the femoral head-neck fragment and the lag screw/helical blade from sliding further laterally, thereby maintaining an almost normal neck length and neck-shaft angle.

However, the lateral telescoping along the axial direction of lag screw/helical blade slippage of the femoral head-neck fragments deserves surgeons' full attention [14]. Some researchers believe that secondary stability following slippage of the femoral head-neck fragment is an important factor related to bone reunion.

Secondary stability depends on the contact between the femoral head-neck fragment and the femoral shaft fragment or the contact between the femoral head-neck fragment and the intramedullary nailing system. In a preliminary study, we proposed the usefulness of positive support for fracture reduction. By increasing the contact between the fragments, the lateral slippage of the femoral head-neck fragment can be reduced [13].

In this study, we found only one free defect fragment in the anterior region. Therefore, the anteromedial region could be considered as the most stable contact area between the femoral head-neck fragment and femoral shaft fragment. As shown by the fracture line distribution, the anteromedial region was also the region with the most concentrated support lines. The contact between femoral head-neck fragments and femoral shaft fragment could rely on the cortex in the anteromedial region. Distribution of the bone defects indicated that most defects were located in the posteromedial region and that the lesser trochanter fragments rarely affected the anteromedial region.

Sharma et al. concluded that the medial size of the lesser trochanter fragment was 1.09 cm (SD: 0.33 cm), about 36% (SD: 10%) of the posterior wall defect [15]. Our results showed that the width of the defect (Dw) was 21.5 mm (SD: 6.1 mm, range: 10–40 mm), 56.3% (SD: 13.7%, range: 27.5–100%) of the medial wall, and hence larger than that reported previously.

This is possibly because the previous study only focused on the shape of the trochanter itself. The free fragments between the lesser trochanter and the anteromedial cortex were neglected, which should be counted as the defect area. Another likely reason is that the measurement direction was not perpendicular to the femoral neck axis.

Although the average width of the defect is 56.3% of the medial wall, in 73% cases (43/59), defects were still located behind the neck axis. The average distance from the anterior edge of the defect area to the femoral neck axis was 3.6 mm (SD: 5.7 mm, range: -15 to 17 mm).

Based on the above data, we believe that anterior cortical contact is the key to resist the sliding of the femoral head-neck fragments.

### 4.4. Lesser Trochanter

The fixation of the lesser trochanter for the unstable pertrochanteric fracture is still debatable. Some researchers believe that fixation of the lesser trochanter is unnecessary, while others recommend fixation to provide posteromedial support. Some surgical procedures have been proposed for the reduction of the lesser trochanter, such as nailing or cable bundling [16]. We divided the lesser trochanter fragments into three types: maintaining a continuation with the greater trochanter (19 cases, 32.20%), separated but intact lesser trochanter fragments (25 cases, 42.37%), and comminution of the lesser trochanter to >3 pieces (15 cases, 25.42%). We believe that fixation of the lesser trochanter is essential for the first two types, but reduction fixation is very difficult to perform in the case of the comminuted lesser trochanter. Therefore, the preoperative observation and virtual fracture reduction are important to better understand the fracture morphology.

In patients with three-part fractures of the greater trochanter, the lesser trochanter was preserved at the side of the femoral shaft. According to the EJ classification, this type of fracture is considered unstable. However, we found through observation that the medial wall (anteromedial and posteromedial) remained intact. Therefore, the fracture should be relatively stable in internal fixation, especially with intramedullary fixation.

### 4.5. Pertrochanteric Crest (in the Back View)

Fracture lines in the pertrochanteric crest usually indicate separation of the lesser and greater trochanters. EL classification does not include the classification of the fragments in the back. Sharma et al. analyzed the morphology of the type A2 greater trochanter fracture in 50 cases by using CT scan and classified the fragments in the back into two types: a banana-shaped fragment with continuation of the lesser and greater trochanters and separate fragments with separation of the lesser and greater trochanters [15]. Among our patients, 17 (28.81%) had intact banana-shaped fragments, and 42 (71.19%) showed separation of the lesser and greater trochanters. This finding is similar to that of Sharma et al. with the fracture lines mainly distributed in the medial half. Moreover, the junction between the pertrochanteric crest and base of the femoral neck was the site of frequent occurrence of separate fracture fragments. This may be probably because of the large backward force acting on the femoral head-neck fragments.

### 4.6. Greater Trochanter

Fracture lines were mainly found anterior to the apex of the greater trochanter, while the posterior part remained more intact. The fracture lines posteriorly extended along the greater trochanter spine, rarely affecting the lateral wall. In our study, only one patient with a type A2 fracture was associated with damage of the lateral wall. Of 18 cases of fracture lines passing through the lateral wall, 17 showed fracture lines extending transversely towards the front, thus affecting the integrity of the pertrochanteric line. This case was reassigned as a type A3 fracture.

### 4.7. Lateral Wall

We noted 10 cases of fracture lines in the lateral wall (16.95%). Among all cases, the fracture lines in OTA 31-A2 were mostly found in the margin of the lateral wall. The femoral body was basically intact, and the stability was hardly affected. Type A3 fractures may lead to loss of stability of the lateral wall. For those with fractures in the posterior margin of the lateral wall, DHS can be placed anteriorly to provide adequate lateral support.

### 4.8. Pertrochanteric Line (in the Front View)

Eight cases (13.56%) had separate fracture fragments in this region. For the remaining cases, the separate fracture fragments were found in the junction between the femoral head-neck fragments and femoral shaft (support lines). Fracture reduction in this region is rarely discussed in existing literature. Tsukada et al. found that patients with anterior cortex injuries were more likely to experience internal fixation failure [17]. Considering the slippage direction of the femoral head-neck fragments, the support in this region deserves full attention. Although the bone cortex is relatively thin in this region, it has a large contact area and abundant cancellous bone, which can play an important part in early bone union and weight bearing in pertrochanteric fractures.

### 4.9. Limitations

The number of cases included in this study is still relatively small; increasing the sample size may more accurately estimate the distribution of fracture lines. This study only analyzed the A2 subtypes of pertrochanteric fractures, and the characteristics of the main fracture fragments of other subtypes needed to be further explored.

## 5. Conclusions

Our study provided new insights into surgical reduction and fixation strategies and demonstrated the most common fracture patterns encountered during surgery. The integrity of the anteromedial cortex should be considered in the internal fixation of femoral trochanteric fractures. These morphological characteristics could be used to form postoperative cortical contact and improve stability of the fixation. Hence, 3D mapping technology can help establish a typical fracture model and improve doctors' understanding of fracture characteristics.

## Figures and Tables

**Figure 1:** Reconstruction and reduction: (a) volume rendering; (b) surface reconstruction; (c) reduction; (d) medial wall width (Mww, red), defect width (Dw, yellow), distance between defect and neck axis (Dd, green), connect medial wall width (Cmww, orange); (e) registration; (f) fracture line drawing (red curve); (g) fracture location (black area) support line (red curve).

**Figure 2:** Fracture line superimpose: (a) medial view; (b) posterior view; (c) lateral view; (d) anterior view; (e) top view; (f) posteromedial view (less trochanteric).

**Figure 3:** Fracture line 3D heat mapping: (a) medial view; (b) posterior view; (c) lateral view; (d) anterior view; (e) top view; (f) posteromedial view (less trochanteric).

**Figure 4:** Fracture defect area location 3D mapping: (a) medial view; (b) posterior view; (c) lateral view; (d) anterior view; (e) top view; (f) posteromedial view (less trochanteric).

**Figure 5:** Support line mapping: (a) support line distribution (anteromedial view); (b) 3D heat mapping.

## Data Availability

All the data are available if qualified authors apply for them.
